# Automatic Optic Disc Segmentation Based on Modified Local Image Fitting Model with Shape Prior Information

**DOI:** 10.1155/2019/2745183

**Published:** 2019-03-14

**Authors:** Yuan Gao, Xiaosheng Yu, Chengdong Wu, Wei Zhou, Xiaoliang Lei, Yaoming Zhuang

**Affiliations:** ^1^College of Information Science and Engineering, Northeastern University, Shenyang, Liaoning 110819, China; ^2^Faculty of Robot Science and Engineering, Northeastern University, Shenyang, Liaoning 110819, China

## Abstract

Accurate optic disc (OD) detection is an essential yet vital step for retinal disease diagnosis. In the paper, an approach for segmenting OD boundary without manpower named full-automatic double boundary extraction is designed. There are two main advantages in it. (1) Since the performances and the computational cost produced by iterations of contour evolution of active contour models- (ACM-) based approaches greatly depend on the initialization, this paper proposes an effective and adaptive initial level set contour extraction approach using saliency detection and threshold techniques. (2) In order to handle unreliable information generated by intensity in abnormal retinal images caused by diseases, a modified LIF approach is presented by incorporating the shape prior information into LIF. We test the effectiveness of the proposed approach on a publicly available DIARETDB0 database. Experimental results demonstrate that our approach outperforms well-known approaches in terms of the average overlapping ratio and accuracy rate.

## 1. Introduction

Optic disc (OD) is a bright yellowish approximately circular or oval-shaped object in the retinal images [1], as shown in Figure 1.

Accurate OD localization and segmentation play an important role in retinal image analysis and eye diseases diagnosis. For instance, the localization of the OD is a crucial step for fovea detection, vessel tracking, measurement, and automated diabetic retinopathy (DR) screening [2]. Meanwhile, the segmentation of the OD can be used for diagnosing other diseases including glaucoma, papilledema, hypertensive retinopathy, and neovascularization of the disc (NVD) [3, 4]. However, in many real applications, there are some challenging problems for OD segmentation due to the complex OD appearance caused by some anomalies, such as myelinated nerve fibers, peripapillary atrophy (PPA), blood vessels covered, and poor image quality. Hence, many scholars have been proposing a series of approaches to improve the precision of OD boundary extraction. These approaches can be divided into four categories including classification-based [5–9], template-based matching [10–17], morphology-based [18–20], active contour models- (ACM-) based approaches [15, 21–24].

Plenty of classification-based OD boundary extraction methods have been presented by Cheng et al. [5], Dutta et al. [6], Tan et al. [7], and Zhou et al. [8, 9]. They utilized image pixel-level features or superpixel-level features extracted from retinal fundus images to segment OD. However, these approaches are easy to be influenced by sample size. Namely, the segmentation results of OD have a larger bias if there is only a small amount of training data. Besides, it is also time consuming when dealing with a large amount of training data.

Template-based matching methods consider the shape prior information of the OD, i.e., the circular or elliptical shape, to match the edge maps extracted from retinal fundus images [10–17]. However, these methods always fail to detect the ODs with varied shapes.

Some morphology techniques are used to extract OD boundary, e.g., Reza et al. [18] and Welfer et al. [19]. In these approaches, the shape and bright of the OD are modeled by some morphology techniques. Nevertheless, the main disadvantage of these approaches is that bright lesions can affect their performance.

Srivastava et al. [20] applied a deep neural network composed of (unsupervised) stacked autoencoders followed by a supervised layer to distinguish OD from retinal fundus images. But it cannot deal well with the problem when the PPA is very similar to the OD.

Compared with the aforementioned approaches, ACM will obtain an excellent OD segmentation result due to the combination of the profound mathematical properties and prior knowledge of the OD. Hence, ACM-based approaches have become the most promising technique to detect the OD boundary [25]. Lee and Brady [21] firstly proposed a gradient vector flow (GVF) base active contour model for extracting the optic disc boundary with a fixed size initial contour followed by reducing the effect produced by high gradient at vessel locations. Mendels [22] presented a novel active contour approach using the gradient vector-flow-driven contour initialized manually to determine the OD boundary after preprocessing the image based on local minima detection and morphological filtering. A modified version of the conventional level-set method proposed by Wong et al. [15] is used to obtain the OD boundary with a constant scale initial contour from the red channel, and the contour is subsequently smoothened by strictly fitting a ellipse. Yu et al. [23] applied a fast, hybrid level set model, in which the deformable contour is driven by the local edge vector and the region information converging to the true optic disc boundary based on fixed size initial contour determined by experience. A variational-level set deformable model designed by Esmaeili et al. [24] has higher convergence property and better computational efficiency compared with other segmentation active contour models when extracting the OD boundary with an empirical estimation initial contour around the detected OD center. These ACM-based methods can accurately segment ODs with strong boundary, but they are always influenced by intensity inhomogeneities and blood vessels occlusion which are highly sensitive to interferences around the boundary, especially for bright lesions adjacent to the boundary of ODs, reducing their performance.

Seen from the above-mentioned OD detection methods, although the exiting ACM-based approaches can achieve better performance than classification-based approaches [5–9], template-based matching approaches [10–17] and morphology-based [18–20], most of ACM [15, 21–24] evolving the contour using the imprecise initial contour which is labeled by hand or is set based on fixed size. It not only reduces the performance for ACM but also generates the expensive computational cost. Besides, these ACM-based methods are misguided by unreliable information generated by intensity for extreme situation in abnormal retinal images caused by diseases, e.g., blurry OD boundary, bright peripapillary atrophy interference, and thick blood vessel coverage. They also need to remedy the insufficient information lost through image preprocessing which has been changed along with the different segmentation methods, making the key information lost, and have a complex operation. To address these issues, this paper proposes a novel approach by combining the local image fitting energy and shape prior information to extract OD boundary. The main contributions are as follows: (1) an automatic and robust adaptive initial level set contour extraction method by combining saliency detection and threshold techniques is designed to achieve the optimized contour evolution. (2) A novel ACM-based approach named local image fitting model with oval-shaped constraint (LIFO) is presented, which integrates the model with oval-shaped constraint into a united framework remedying the deficiency of only considering the information of intensity.

## 2. Methods

### 2.1. Optic Disc Localization

In this paper, we use our previous work [26] to locate the OD. In [26], a series of OD candidates can be firstly extracted using morphological opening by reconstruction. Then, a set of features are used to distinguish the true optic disc from the nonoptic disc candidates (for more details, refer [26]).

### 2.2. Optic Disc Segmentation

#### 2.2.1. Rough Boundary Extraction of the OD

Based on the cropped region of interest around optic disc, we can further extract the optic disc boundaries. Since the contour initialization is the basic step to initialize the proposed active contour model, we propose a novel and robust contour initialization approach by combining saliency detection and threshold techniques together in this paper. The details are as follows.

Since the optic disc region is usually of a brighter pallor than the surrounding retinal areas, it can be regarded as a salient objective in retinal fundus images. Recently, inspired by saliency detection technique which aims at finding out the most important part of an image, we adopt a cellular (i.e., superpixel) automata-based saliency detection approach [27] by taking both global color and spatial distance matrices into consideration to contour initialization. First, cellular automata-based saliency detection approach [27] is done on the tailored image.  Figure 2(a) is the obtained saliency map in which the corresponding output saliency value of each superpixel is continuous between 0 and 1, as shown in Figure 2(b). Then, a mean filter is found to be a good choice [5] which is then applied on the saliency map to achieve smoothed map values, as shown in Figure 2(c). Next, the smoothed map values are then used to acquire the binary decisions for all the pixels with a threshold. In our experiment, we obtain the threshold by Otsu's thresholding and assign 1 and 0 to optic disc and nonoptic disc. After we obtain binary decisions for all the pixels, the values with 1 are regarded as object (optic disc) and 0 as background. Finally, the largest connected object (i.e., the connected region with the largest number of the pixels) can be obtained through morphological operation, as shown in Figure 2(d). And its boundary is used as the raw estimation of the optic disc, i.e., the optic disc initial contour in green, as shown in Figure 2(e).

#### 2.2.2. Accurate Boundary Curve Extraction

Considering the intensity inhomogeneity is a frequently occurring phenomenon in the optic disc region [28]; the optic disc boundary extracted by general segmentation methods is usually inaccurate due to intensity inhomogeneity caused by imperfection of image devices or illumination variations. In order to deal with this problem, the local image fitting (LIF) model presented by Zhang et al. [28] is introduced; it defines local image fitting energy in a variational formulation which incorporates local intensity information into the active contour model. The LIF model can be described as follows:

(1) $$\begin{array}{c} E^{\text{LIF}}=\frac{1}{2}\int_{\Omega }{\left|I-I^{\text{LFI}}\right|}^{2}\;dx, \end{array}$$

where

(2) $$\begin{array}{c} I^{\text{LFI}}=m_{1}H\left(\phi \right)+m_{2}\left(1-H\left(\phi \right)\right), \end{array}$$

(3) $$\begin{array}{c} m_{1}=\text{mean}\left(I\in \left(\left\{\left.x\in \Omega \right|\phi \left(x\right)<0\right\}\cap W\left(x\right)\right)\right), \end{array}$$

(4) $$\begin{array}{c} m_{2}=\text{mean}\left(I\in \left(\left\{\left.x\in \Omega \right|\phi \left(x\right)>0\right\}\cap W\left(x\right)\right)\right), \end{array}$$

where *I* denotes an input image; *I* ^LFI^ is a local fitted image (LFI) formulation, *m*_1_ and *m*_2_ are, respectively, defined as local mean near the point *x* described by equations (3) and (4). *x* is the variable to express the location information of pixel for global, *Ω* is the image domain, *ϕ* is a level set function, *H*(*ϕ*) is the Heaviside function, and *W*(*x*) is a rectangular window function defined in [28].

Considering that the fundamental anatomical structure of the OD, e.g., it is a bright approximately circular or elliptic region, we can regard the anatomical structure as a shape prior constraint and take it into our model. In this paper, we incorporate both the smoothing item and an oval-disc prior constraint into LIF model, and the novel model named local image fitting model with oval-shaped constraint (LIFO) is proposed for OD boundary extraction. The model can remedy insufficiency of LIF, such as the LIF model will fail to extract the OD boundary with some blood vessels as shown in Figure 3(b). Seen from the result in Figure 3(c), the novel model overcomes the influence of blood vessels and intensity inhomogeneities achieving a precise OD boundary extraction of Figure 3(a).

Seen from the above results, it is necessary to introduce the smoothing item and shape prior information into LIF model aiming to acquire a whole boundary of the OD. They can be formulated as follows:

(5) $$\begin{array}{c} E^{\text{prior}}=E^{\text{smooth}}+E^{\text{ellipse}}, \end{array}$$

(6) $$\begin{array}{c} E^{\text{smooth}}=\nu \int_{\Omega }\delta \left(\phi \right)\left|\nabla \phi \right|\;dx, \end{array}$$

(7) $$\begin{array}{c} E^{\text{ellipse}}=\frac{1}{2}\alpha \int_{\Omega }{\left(H\left(\phi \right)-H\left(\phi_{\text{e}}\right)\right)}^{2}\;dx, \end{array}$$

where

(8) $$\begin{array}{c} \phi_{\text{e}}=1-\sqrt{\frac{{\left[\left(x_{i}-x_{\text{e}}\right)\cos\;\theta_{\text{e}}+\left(y_{i}-y_{\text{e}}\right)\sin\;\theta_{\text{e}}\right]}^{2}}{a_{\text{e}}^{2}}+\frac{{\left[-\left(x_{i}-x_{\text{e}}\right)\sin\;\theta_{\text{e}}+\left(y_{i}-y_{\text{e}}\right)\cos\;\theta_{\text{e}}\right]}^{2}}{b_{\text{e}}^{2}}}\text{ ,} \end{array}$$

where ∇ is the gradient operator; *δ*(*ϕ*) is the smooth Dirac function; *x*_*i*_ and *y*_*i*_ are, respectively, *x*-coordinate and *y*-coordinate for global pixel information *x*; *x*_e_ and *y*_e_ are oval center coordinates; *θ*_e_ is the angle of rotation; *a*_e_ denotes scaling factors of semimajor axis length; and *b*_e_ is defined as semiminor axis length. *ϕ*_e_ is the level set based on ellipse shape. Both of them are constantly changed with the curve evolution. In fact, the purpose for calculating equation (5) is to acquire the level set *ϕ* which is similar to *ϕ*_e_. The novel model named LIFO can be obtained by combining equations (1) and (5) into a unified framework:

(9) $$\begin{array}{c} E^{\text{LIFO}}=\left(E^{\text{LIF}}+E^{\text{prior}}\right), \end{array}$$

(10) $$\begin{array}{c} E=\frac{1}{2}\int_{\Omega }{\left|I-I^{\text{LFI}}\right|}^{2}\;dx+\nu \int_{\Omega }\delta \left(\phi \right)\left|\nabla \phi \right|\;dx+\frac{1}{2}\alpha \int_{\Omega }{\left(H\left(\phi \right)-H\left(\phi_{\text{e}}\right)\right)}^{2}\;dx, \end{array}$$

where *α* is the constraint coefficient for ellipse which decides the weight of elliptic constraint and *v* is the coefficient of the weighted length of zero level curve of *ϕ*.

There are three terms in the LIFO model (equation (10)) and each of them has its unique function to deal with different problems in OD boundary extraction. The first term *E* ^LIF^ is used to deal with the commonly occurred phenomenon in the optic disc regions that are always influenced by intensity inhomogeneity. The second term is the smooth item, which is used to handle drastic protuberance and sunken for evaluated contours by penalizing arc length of zero level contour of *ϕ*. The third term is the oval-shaped constraint term for ensuring the evaluated contour which can satisfy with the physical anatomical structure of optic disc, reducing the impact of complex environments. The LIFO model can be solved by the standard gradient descent method [28]. After a series of calculations, the solution is obtained in Appendix.

The flow diagram for segmentation of the OD is as follows:

1. Initialization: *v*=0.0001 × 255 × 255, *α*=1.0, *x*_e_=width/2, *y*_e_=height/2, *θ*_e_=0, $a_{\text{e}}=\sqrt{{\text{width}}^{2}+{\text{height}}^{2}}/8$, $b_{\text{e}}=\sqrt{{\text{width}}^{2}+{\text{height}}^{2}}/8$ (the width and the height are, respectively, the width and the height of the cropped region for the original image), the level set functions *ϕ* ^*l*^=*ϕ* ^0^, *ϕ*_e_^*l*^=*ϕ*_e_^0^, and *l* and *r* denote iterations.
2. Update *m*_1_ and *m*_2_, respectively, using equations (3) and (4).
3. Update *I* ^LFI^ using equation (2).
4. Using the standard gradient descent method, evolve the parameters of elliptical level set of the OD including *x*_e_, *y*_e_, *θ*_e_, *a*_e_, *b*_e_ according to equations (A.1)–(A.5); if *x*_e_^*r*^, *y*_e_^*r*^, *θ*_e_^*r*^, *a*_e_^*r*^, *b*_e_^*r*^ satisfy the stationary condition, then stop; else *r*=*r*+1 and return to Step 4.
5. Update *ϕ*_e_^*l*^ using equation (8).
6. Evolve the level set functions, according to equation (A.6). If *ϕ* ^*l*^ satisfy the stationary condition, stop; otherwise, *l*=*l*+1 and return to Step 2.

## 3. Experimental Results

In this section, the public Standard Diabetic Retinopathy Database “Calibration Level 0” (DIARETDB0) [29] and the public dataset of retinal images namely DRISHTI-GS [30] are applied to verify the availability of our method. The DIARETDB0 and DRISHTI-GS are available and can be downloaded from the web pages http://www.it.lut.fi/project/imageret/diaretdb0/ and http://cvit.iiit.ac.in/projects/mip/drishti-gs/mip-dataset2/Home.php._The_DIARETDB0 database is made up of 130 RGB color fundus images of which 20 are normal and 110 are abnormal (illness) with the fixed 1500 × 1152 resolution and 50° field of view. The ground truth is collected from two ophthalmologists. The final ground truth is acquired by averaging boundary results extracted from two ophthalmologists. The DRISHTI-GS dataset totally has 101 images of which 31 are normal and 70 are abnormal (illness). These images are produced with 30° degree field of view and have a resolution of 2896 × 1944. For each image, the OD is correctly marked by four glaucoma experts. To compensate for interobserver marking variations, we also derive a majority voting manual marking as the final ground truth indicating that agreement among at least three experts [30] to qualitatively evaluate the proposed method.

Seen from Figure 4, compared with different contour evolution approaches using adaptive initial contour and different initial circular contours based on the fundamental anatomical structure of the OD, there are some advantages for the proposed approach. First, most of ACM-based approaches are sensitive to the initialization of the contour [32]. However, the proposed initial contour can better guide the motion of the active contour since it is close to the ground truth of OD boundary. Second, the adopted initial contour which is near the OD boundary can reduce iterations of contour evolution. Therefore, it can reduce the computational cost [33, 34]. Furthermore, compared with the original LIF [28], our approach is more robust to the influence caused by the blood vessels due to the fact that the oval-shaped constraint is incorporated into our model.

The criterion is adopted to further assess the availability of LIFO model with different initial contours; it is considered that the overlapping ratio *T* which is computed based on the overlapping area between the true optic disc region in the ground truth and the detected optic disc region is no less than 75% for successful segmentation in terms of [11]. The accuracy ratio is the percentage ratio of successfully classified images to the total number of images. The overlapping ratio *T* is defined as

(11) $$\begin{array}{c} T=\frac{\text{area}\left(G\cap D\right)}{\text{area}\left(G\cup D\right)}, \end{array}$$

where *G* and *D* are, respectively, the area of ground truth and the area extracted by the methods.  Table 1 shows accuracy rate acquired by different initial contours.

Seen from Table 1, the proposed method achieves the best segmentation result with adaptive initial contour, and the accuracy rate is, respectively, 96.30% and 96.10% on the DIARETDB0 database and the DRISHTI-GS database.

In order to better verify the effectiveness of the proposed method, we compare our method with some related and newest approaches for segmentation in medical image processing area such as Hough transform method [31], modified radial symmetry method (MRS) [35], GVF method [36], Chan-Vese (CV) ACM [37], LIF ACM [28], and LSACM ACM [38]. The different segmentation results obtained by all five methods from retinal images are given in Figure 5, in which the green line denotes the ground truth obtained from the experts' marking and the red line represents some segmentation results extracted by different approaches. The examples of the OD having peripapillary atrophy are shown in the first three columns, and the OD with irregular shape and high gradient variations is shown in the fourth column. The Hough transform and the GVF model fail to extract the whole OD boundary due to the fact that they are sensitive to the varying of local gradient. Although MRS can achieve more accurate result than Hough transform, it ignores that the OD is an approximately circular or elliptic region rather than rigid circular region. However, the CV model models image as piecewise constant function which fails to handle intensity inhomogeneity in retinal image, and thereby achieves unsatisfactory segmentation result. Although the LIF model can deal with these local gradient variations well compared to GVF and Hough transform and reduce the influence of intensity inhomogeneity because of considering local intensity information; it is severely influenced by blood vessel covering the OD surface. The LSACM model also can handle the intensity inhomogeneity and achieve more integrated OD boundary compared to the LIF model because it models the objects as Gaussian distributions of different means and variances; however, it is defeated by blood vessels and PPA obtaining a deficient segmentation result. Seen from the aforementioned methods, our method performs better and captures the whole OD boundary, which overcomes the influence caused by intensity inhomogeneity, PPA, and blood vessels. The fifth column shows a successful result segmented by LIFO model in blurry OD region with smooth transition boundary. This is mainly due to the fact that the prior shape information in some regions is a stronger cue than the intensity information. Therefore, combining the prior information and intensity information together can obtain the smooth and precise OD boundary.

Table 2, respectively, shows the average overlapping ratio and accuracy rate acquired by different models.

As seen from Table 2, we can clearly see that our method can get a better performance from DIARETDB0/DRISHTI-GS compared with other methods in terms of average overlapping ratio 66.59%/65.61% and accuracy rate 96.30%/96.10% for successful segmentation in retinal images including normal and abnormal (illness). The average overlapping ratio of segmentation obtained by proposed method in retinal image for normal/abnormal is 67.33% and 66.25%/65.53% and 64.87%; the accuracy rate of segmentation obtained by the proposed method in retinal image for normal/abnormal is 98.40% and 98.90%/95.90% and 94.90% on the DIARETDB0 and the DRISHTI-GS, respectively.

Besides, we also use an important evaluation metric *F*-score (*F*) which is the harmonic mean of precision and recall between the achieved boundary by the method and ground truth to test the performance of the proposed model. The pixelwise precision and recall values are, respectively, defined as

(12) $$\begin{array}{c} \text{precision}=\frac{\text{tp}}{\text{tp}+\text{fp}},\\ \text{recall}=\frac{\text{tp}}{\text{tp}+\text{fn}}, \end{array}$$

where true positive (tp) indicates the number of pixels in the coverage areas between the ground truth and achieved segmented area by the methods; false positive (fp) expresses the number of pixels in the area where the pixel is classified only in the segmented area by the methods and is excluded belonging to the ground truth; false negative (fn) is the number of pixels in the area where a pixel is classified only in the ground truth and is excluded belonging to the segmented area by the methods. Then, the single performance measure, namely, *F*-score (*F*) is computed and defined as

(13) $$\begin{array}{c} F=2\frac{\text{precision}\cdot \text{recall}}{\text{precision}+\text{recall}}. \end{array}$$

The value of *F*-score always lies between 0 and 1 and will be high if the performance of method is good.

Table 3 depicts the quantitative assessment for segmentation results in terms of the *F*-score. The best and the worst achieved by the proposed method are, respectively, the best case and the worst case for fundamental results of the optical disc from the DIARETDB0 and the DRISHTI-GS. Seen from Table 3, it can be inferred that our method has a significant improvement in the segmentation results compared to others methods.

## 4. Conclusions

In this paper, we design a strategy to accurately segment OD boundary without manpower. First, an automatic and robust adaptive initial level set contour extraction method consisting of saliency detection and threshold techniques is presented for making the contour evolution. Then, in order to remedy the deficiency that only considers the intensity and ignores the prior information for OD shape, an excellent local image fitting model with oval-shaped constratint (LIFO) is presented to extract the whole and precise OD boundary. Comparing with the original LIF model only based on intensity information, the LIFO model uses both of the intensity information and shape information which has the following advantages. First, the original model is easily influenced by PPA, blood vessels, and noise due to only considering the intensity information. On the contrary, the proposed model can overcome these issues by using both of the intensity information and the shape prior information without any preprocessing. Second, the proposed model introduces the shape prior information based on the physical anatomical structure of the optic disc, and it can extract the whole boundary of the optic disc especially for the irregular shape of the optic disc. The experimental results demonstrate the availability of the proposed method. Now, the deep learning has attracted attention and achieves a good performance when the number of training samples is enough. However, it is hard to collect enough data in medical field such as the retinal fundus images, which will greatly reduce the performance of model. That is the main reason why we did not employ the deep learning technique to segment the optic disc and optic cup. In the future, we will try to use the deep learning approaches on the larger database.

## Figures and Tables

**Figure 1:** Major structures of the optic disc. Red line: the optic disc boundary.

**Figure 2:** Contour initialization. (a) Cropped ROI around optic disc; (b) saliency detection result; (c) smoothed image of (b); (d) the largest connected object; (e) optic disc initial contour in green.

**Figure 3:** The result of OD boundary extraction obtained by LIF model and LIFO model, respectively; the ground truth is marked with a green line.

**Figure 4:** The comparisons for different segmentation models with different initial contours and Hough transform method. They, respectively, show the comparison results based on adaptive initial contour and manual initial circular contour drawing outside of the OD, inside of the OD, and intersect of the OD. The ground truth is marked with a green line. (a) Initial level set contour. (b) Presented LIFO. (c) LIF [28]. (d) Hough transform [31].

**Figure 5:** OD segmentation results: (a) original image with the ground truth; (b) adaptive initialized contour; (c) Hough transform results [31]; (d) MRS results [35]; (e) GVF model results [36]; (f) CV model results [37]; (g) LIF model results [28]; (h) LSACM model results [38]; (i) proposed LIFO model results. Green color indicates boundary marked by the expert and red color indicates achieved boundary by a method.

**Table 1:** Performance measurement based on overlapping areas between different initial contours on the DIARETDB0 database and the DRISHTI-GS database.

Initial contour	Accuracy rate (DIARETDB0) (%)	Accuracy rate (DRISHTI-GS) (%)
Contour intersecting the OD	94.50	94.10
Contour within the OD	94.80	94.50
Contour outside the OD	95.10	95.30
Adaptive contour	96.30	96.10

**Table 2:** Performance measurement based on overlapping areas between the proposed approach and other segmentation approaches on the DIARETDB0 database and DRISHTI-GS database.

	Average overlapping ratio (DIARETDB0) (%)	Accuracy rate (DIARETDB0) (%)	Average overlapping ratio (DRISHTI-GS) (%)	Accuracy rate (DRISHTI-GS) (%)
Hough [31]	61.42	89.60	60.55	88.10
MRS [35]	61.96	90.80	60.81	88.60
GVF [36]	63.66	92.80	61.86	91.30
CV [37]	55.15	86.10	55.15	85.30
LIF [28]	63.89	93.10	63.02	91.70
LSACM [38]	64.24	93.90	63.91	93.50
Ours (LIFO)	66.59	96.30	65.61	96.10
Normal	67.33	98.40	66.25	98.90
Abnormal	65.53	95.90	64.87	94.90

**Table 3:** Performance measurement based on *F*-score between the proposed approach and other segmentation approaches on the DIARETDB0 database and DRISHTI-GS database.

Methods	*F*-score (average) (DIARETDB0)	*F*-score (average) (DRISHTI-GS)
Hough [31]	0.853	0.841
MRS [35]	0.865	0.859
GVF [36]	0.885	0.882
CV [37]	0.792	0.786
LIF [28]	0.915	0.908
LSACM [38]	0.937	0.919
Ours(LIFO)	0.951	0.946
Best	0.986	0.990
Worst	0.658	0.646

## Data Availability

The data used to support the findings of this study are available from the corresponding author upon request.

## Appendix

The LIFO model can be solved by the standard gradient descent method [28]. After a series of calculations, the solution is obtained as follows:

(A.1) $$\begin{array}{c} \frac{dx_{\text{e}}}{dt}=\alpha \int_{\Omega }\left(H\left(\phi \right)-H\left(\phi_{\text{e}}\right)\right)\delta \left(\phi_{\text{e}}\right)\times {\left(\frac{{\left[\left(x_{i}-x_{\text{e}}\right)\cos\;\theta_{\text{e}}+\left(y_{i}-y_{\text{e}}\right)\sin\;\theta_{\text{e}}\right]}^{2}}{a_{\text{e}}^{2}}+\frac{{\left[-\left(x_{i}-x_{\text{e}}\right)\sin\;\theta_{\text{e}}+\left(y_{i}-y_{\text{e}}\right)\cos\;\theta_{\text{e}}\right]}^{2}}{b_{\text{e}}^{2}}\right)}^{-\left(1/2\right)}\left(\frac{\left[\left(x_{i}-x_{\text{e}}\right)\cos\;\theta_{\text{e}}+\left(y_{i}-y_{\text{e}}\right)\sin\;\theta_{\text{e}}\right]\cos\;\theta_{\text{e}}}{a_{\text{e}}^{2}}+\frac{-\left[-\left(x_{i}-x_{\text{e}}\right)\sin\;\theta_{e}+\left(y_{i}-y_{\text{e}}\right)\cos\;\theta_{\text{e}}\right]\sin\;\theta_{\text{e}}}{b_{\text{e}}^{2}}\right)\;dx, \end{array}$$

(A.2) $$\begin{array}{c} \frac{dy_{\text{e}}}{dt}=\alpha \int_{\Omega }\left(H\left(\phi \right)-H\left(\phi_{\text{e}}\right)\right)\delta \left(\phi_{\text{e}}\right)\times {\left(\frac{{\left[\left(x_{i}-x_{\text{e}}\right)\cos\;\theta_{\text{e}}+\left(y_{i}-y_{\text{e}}\right)\sin\;\theta_{\text{e}}\right]}^{2}}{a_{\text{e}}^{2}}+\frac{{\left[-\left(x_{i}-x_{\text{e}}\right)\sin\;\theta_{\text{e}}+\left(y_{i}-y_{\text{e}}\right)\cos\;\theta_{\text{e}}\right]}^{2}}{b_{\text{e}}^{2}}\right)}^{-\left(1/2\right)}\left(\frac{\left[\left(x_{i}-x_{\text{e}}\right)\cos\;\theta_{\text{e}}+\left(y_{i}-y_{\text{e}}\right)\sin\;\theta_{\text{e}}\right]\sin\;\theta_{\text{e}}}{a_{\text{e}}^{2}}+\frac{\left[-\left(x_{i}-x_{\text{e}}\right)\sin\;\theta_{\text{e}}+\left(y_{i}-y_{\text{e}}\right)\cos\;\theta_{\text{e}}\right]\cos\;\theta_{\text{e}}}{b_{\text{e}}^{2}}\right)dx, \end{array}$$

(A.3) $$\begin{array}{c} \frac{d\theta_{\text{e}}}{dt}=\alpha \underset{\Omega }{\int }\left(H\left(\phi \right)-H\left(\phi_{\text{e}}\right)\right)\delta \left(\phi_{\text{e}}\right)\times {\left(\frac{{\left[\left(x_{i}-x_{\text{e}}\right)\cos\;\theta_{\text{e}}+\left(y_{i}-y_{\text{e}}\right)\sin\;\theta_{\text{e}}\right]}^{2}}{a_{\text{e}}^{2}}+\frac{{\left[-\left(x_{i}-x_{\text{e}}\right)\sin\;\theta_{\text{e}}+\left(y_{i}-y_{\text{e}}\right)\cos\;\theta_{\text{e}}\right]}^{2}}{b_{\text{e}}^{2}}\right)}^{-\left(1/2\right)}\left(\frac{-\left[\left(x_{i}-x_{\text{e}}\right)\cos\;\theta_{\text{e}}+\left(y_{i}-y_{\text{e}}\right)\sin\;\theta_{\text{e}}\right]\left[-\left(x_{i}-x_{\text{e}}\right)\sin\;\theta_{\text{e}}+\left(y_{i}-y_{\text{e}}\right)\cos\;\theta_{\text{e}}\right]}{a_{\text{e}}^{2}}+\frac{\left[\left(x_{i}-x_{\text{e}}\right)\cos\;\theta_{\text{e}}+\left(y_{i}-y_{\text{e}}\right)\sin\;\theta_{\text{e}}\right]\left[-\left(x_{i}-x_{\text{e}}\right)\sin\;\theta_{\text{e}}+\left(y_{i}-y_{\text{e}}\right)\cos\;\theta_{\text{e}}\right]}{b_{\text{e}}^{2}}\right)\;dx, \end{array}$$

(A.4) $$\begin{array}{c} \frac{da_{\text{e}}}{dt}=\alpha \int_{\Omega }\left(H\left(\phi \right)-H\left(\phi_{\text{e}}\right)\right)\delta \left(\phi_{\text{e}}\right)\times {\left(\frac{{\left[\left(x_{i}-x_{\text{e}}\right)\cos\;\theta_{\text{e}}+\left(y_{i}-y_{\text{e}}\right)\sin\;\theta_{\text{e}}\right]}^{2}}{a_{\text{e}}^{2}}+\frac{{\left[-\left(x_{i}-x_{\text{e}}\right)\sin\;\theta_{\text{e}}+\left(y_{i}-y_{\text{e}}\right)\cos\;\theta_{\text{e}}\right]}^{2}}{b_{\text{e}}^{2}}\right)}^{-\left(1/2\right)}\left(\frac{{\left[\left(x_{i}-x_{\text{e}}\right)\cos\;\theta_{\text{e}}+\left(y_{i}-y_{\text{e}}\right)\sin\;\theta_{\text{e}}\right]}^{2}}{a_{\text{e}}^{3}}\right)\;dx, \end{array}$$

(A.5) $$\begin{array}{c} \frac{db_{\text{e}}}{dt}=\alpha \int_{\Omega }\left(H\left(\phi \right)-H\left(\phi_{\text{e}}\right)\right)\delta \left(\phi_{\text{e}}\right)\times {\left(\frac{{\left[\left(x_{i}-x_{\text{e}}\right)\cos\;\theta_{\text{e}}+\left(y_{i}-y_{\text{e}}\right)\sin\;\theta_{\text{e}}\right]}^{2}}{a_{\text{e}}^{2}}+\frac{{\left[-\left(x_{i}-x_{\text{e}}\right)\sin\;\theta_{\text{e}}+\left(y_{i}-y_{\text{e}}\right)\cos\;\theta_{\text{e}}\right]}^{2}}{b_{\text{e}}^{2}}\right)}^{-\left(1/2\right)}\left(\frac{{\left[-\left(x_{i}-x_{\text{e}}\right)\sin\;\theta_{\text{e}}+\left(y_{i}-y_{\text{e}}\right)\cos\;\theta_{\text{e}}\right]}^{2}}{b_{\text{e}}^{3}}\right)dx, \end{array}$$

(A.6) $$\begin{array}{c} \frac{\partial \phi }{\partial t}=v\delta \left(\phi \right)\mathrm{div}\left(\frac{\nabla \phi }{\left|\nabla \phi \right|}\right)+\delta \left(\phi \right)\left(I-I^{\text{LFI}}\right)\left(m_{1}-m_{2}\right)-\alpha \delta \left(\phi \right)\left[H\left(\phi \right)-H\left(\phi_{\text{e}}\right)\right], \end{array}$$

where *x*_e_, *y*_e_, *θ*_e_, *a*_e_, *b*_e_ continually vary along with the changing of information in image and *t* is the time step of the experiment.
